The article "The Complex Regulation of Tanshinone IIA in Rats with Hypertension-Induced Left Ventricular Hypertrophy" was retracted in 2024. Reasons: duplicated images; duplicated data; overlap with earlier publications; original data or images not available.

# The Complex Regulation of Tanshinone IIA in Rats with Hypertension-Induced Left Ventricular Hypertrophy

**DOI:** 10.1371/journal.pone.0092216

**Published:** 2014-03-19

**Authors:** Hui Pang, Bing Han, Tao Yu, Zhen Peng

**Affiliations:** 1 Department of Cardiovascular Medicine, Central Hospital of Xuzhou, Xuzhou Clinical School of Xuzhou Medical College, Affiliated Hospital of Southeast University, Xuzhou, Jiangsu, China; 2 Department of Ultrasonography, Central Hospital of Xuzhou, Xuzhou Clinical School of Xuzhou Medical College, Affiliated Hospital of Southeast University, Xuzhou, Jiangsu, China; University of Milano, Italy

## Abstract

Tanshinone IIA has definite protective effects on various cardiovascular diseases. However, in hypertension-induced left ventricular hypertrophy (H-LVH), the signaling pathways of tanshinone IIA in inhibition of remodeling and cardiac dysfunction remain unclear. Two-kidney, one-clip induced hypertensive rats (n = 32) were randomized to receive tanshinone IIA (5, 10, 15 mg/kg per day) or 5% glucose injection (GS). Sham-operated rats (n = 8) received 5%GS as control. Cardiac function and dimensions were assessed by using an echocardiography system. Histological determination of the fibrosis and apoptosis was performed using hematoxylin eosin, Masson’s trichrome and TUNEL staining. Matrix metalloproteinase 2 (MMP2) and tissue inhibitor of matrix metalloproteinases type 2 (TIMP2) protein expressions in rat myocardial tissues were detected by immunohistochemistry. Rat cardiomyocytes were isolated by a Langendorff perfusion method. After 48 h culture, the supernatant and cardiomyocytes were collected to determine the potential related proteins impact on cardiac fibrosis and apoptosis. Compared with the sham rats, the heart tissues of H-LVH (5%GS) group suffered severely from the oxidative damage, apoptosis of cardiomyocytes and extracellular matrix (ECM) deposition. In the H-LVH group, tanshinone IIA treated decreased malondialdehyde (MDA) content and increased superoxide dismutase (SOD) activity. Tanshinone IIA inhibited cardiomyocytes apoptosis as confirmed by the reduction of TUNEL positive cardiomyocytes and the down-regulation of Caspase-3 activity and Bax/Bcl-2 ratio. Meanwhile, plasma apelin level increased with down-regulation of APJ receptor. Tanshinone IIA suppressed cardiac fibrosis through regulating the paracrine factors released by cardiomyocytes and the TGF-β/Smads signaling pathway activity. In conclusion, our *in vivo* study showed that tanshinone IIA could improve heart function by enhancing myocardial contractility, inhibiting ECM deposition, and limiting apoptosis of cardiomyocytes and oxidative damage.

The article "The Complex Regulation of Tanshinone IIA in Rats with Hypertension-Induced Left Ventricular Hypertrophy" was retracted in 2024. Reasons: duplicated images; duplicated data; overlap with earlier publications; original data or images not available.

## Introduction

Hypertension is a progressive vascular syndrome characterized by continuous increase in arterial blood pressure. It is one of the major risk factors for cardiovascular diseases, and is always complicated with multiple risk factors, impairments in target organs or clinical diseases [1]. In response to the elevated pressure load, the left ventricular (LV) wall thickens as a compensatory mechanism to minimize wall stress. The mechanisms responsible for different grades of severity of left ventricular hypertrophy (LVH) involve not only the pressure load itself, whether it be the severity, duration, or rate of increase of the blood pressure, but also the influences of neurohormones [2], growth factors, cytokines [3] and genetic factors. There is widespread agreement that LVH is defined as an increase in LV mass attributable to wall thickening or chamber dilation [4]. Pathologic features of LVH include an increase in cardiomyocyte size, LV hypertrophy and cardiac fibrosis, which is marked by changes in the quality and quantity of the extracellular matrix (ECM) [5], [6]. LVH one of the most important risk factors results in a worse cardiovascular prognosis. Thus, we suggest that additional clinical benefit from the inhibition of LVH as a potential therapeutic target is as important as the blood pressure control.

Danshen is a crude herbal drug extracted from the dry root and rhizome of Salvia miltiorrhiza Bge (Labiatae) [7]. Tanshinone IIA is one of the main components isolated from Danshen for the treatment of cardiovascular diseases including hypertension [8], cardiac hypertrophy [9], heart failure [10], and myocardial ischemia-reperfusion injury [11]. It can improve heart function [12] by limiting oxidative stress [13], attenuating cardiac fibrosis [14], and inhibiting the hypertrophy and apoptosis of cardiomyocytes. Tanshinone IIA, an ideal cardio-protective agent, can regulate numerous molecular targets including transcription factors, scavenger receptors, ion channels, kinases, pro- and anti-apoptotic proteins, growth factors, inflammatory mediators, microRNA, and others [15]. However, in hypertension-induced hypertrophy, the signaling pathways of tanshinone IIA in inhibition of remodeling and cardiac dysfunction are not fully understood. Our in vivo study was to determine the protective molecular mechanisms from three major respects, reducing apoptosis, inhibiting cardiac fibrosis and decreasing oxidative stress. The molecular mechanisms in apoptosis involve initiator cysteinyl-aspartate proteases (caspases) activation, apoptotic body formation, and cell fragmentation [16]. Some of the paracrine factors released by cardiomyocytes may influence ECM regulation through multiple synergistic paracrine mechanisms [17]. Therefore, we explored the roles of transforming growth factor β1 (TGF-β1) [18] and basic fibroblast growth factor (bFGF) as possible paracrine molecular regulators of this remodeling response.

The article "The Complex Regulation of Tanshinone IIA in Rats with Hypertension-Induced Left Ventricular Hypertrophy" was retracted in 2024. Reasons: duplicated images; duplicated data; overlap with earlier publications; original data or images not available.

## Materials and Methods

### Animals and Reagents

The experimental protocol was approved by the Animal Care and Use Committee of Xuzhou Medical College. Rats were housed in a climate-controlled room. Sterile water and standard chow diet were available ad libitum. Six-week-old male Sprague-Dawley (SD) rats were provided by the Animal Department, Xuzhou Medical College. All of the antibodies, including anti-forkhead box H1 (Foxh1) antibody, anti-c-Myc antibody, anti-p-Smad3 antibody, anti-matrix metalloproteinase 2 (MMP2) antibody, anti-tissue inhibitor of matrix metalloproteinases type 2 (TIMP2) antibody, anti-Bax antibody, anti-Bcl-2 antibody, anti- Caspase-3 antibody and anti-APJ antibody, were purchased from Santa Cruz Biotechnology (Santa Cruz, CA, USA). All other reagent-grade chemicals were purchased from the Sigma- Aldrich Chemical Co. (St. Louis, MO, USA).

### Experimental Designs

Male SD rats (200∼220 g) were subjected to hypertension as described previously [19]. Briefly, a U-shaped silver clip having internal diameter of 0.2 mm was placed around the left renal artery after the rats under 10% chloral hydrate anesthesia. Sham-operated rats underwent a similar procedure without clip of the left renal artery. We performed our analysis on systolic blood pressure (SBP) in unanesthetized rats via noninvasive tail cuff. Four weeks after clipping, if SBP was higher than 160 mmHg, the animals were considered hypertensive. Then the hypertensive rats (n = 32) were randomized to receive tanshinone IIA (5, 10, 15 mg/kg per day) or 5% glucose injection (GS) in a dose matched design. Blood pressure was observed at two weeks intervals following tanshinone IIA therapy. Sham-operated rats (n = 8) received 5% GS as control. Eight weeks later, the animals’ plasma was extracted and heart was removed for use.

### Determination of Cardiac Function

Cardiac function and dimensions were assessed by using an echocardiography system (GE Healthcare Ultrasound, Horten, Norway; 11.5 MHz linear transducer). All measurements were made with the animals under full anesthesia and the body temperature maintained at 36–37°C with the ST-1 homeothermic blanket system. The echocardiography parameters measured were: the left ventricular internal dimension at end diastole (LVIDd), interventricular septal thickness at end diastole (IVSd), left ventricular posterior wall thickness at end diastole (LVPWd), LV fractional shortening (FS%) and ejection fraction (EF%). All parameters were measured five times by the same observer in a blinded method, with the final result the average of the five.

The article "The Complex Regulation of Tanshinone IIA in Rats with Hypertension-Induced Left Ventricular Hypertrophy" was retracted in 2024. Reasons: duplicated images; duplicated data; overlap with earlier publications; original data or images not available.

### Histological Determination of Fibrosis and Apoptosis

Fresh heart ventricles were fixed using 4% paraformaldehyde, dehydrated with alcohol, embedded in paraffin, and cut into 5 mm slices (RM2016, Leica, Wetzlar, Germany). All hearts were embedded in a cross section orientation, and all slices were taken from the cross section at the papillary muscle level of the left ventricles. Three cross sections of each heart were analyzed. From each section, eight areas of hematoxylin eosin and Masson’s trichrome stained slices were randomly selected across the wall thickness to assess the relative fibrosis area (expressed as a percentage of total heart area). Each field was taken at 200 magnification (IX71, Olympus, Tokyo, Japan) and then analyzed using the Adobe ImageReady 7.0.1 software (Adobe Systems, San Jose, CA).

Apoptosis assays were carried out using the terminal deoxynucleotidyl transferase dUTP nick- end labeling (TUNEL) kit (ZSGB-BIO, Beijing, China) and the protocol recommended by the manufacturer. The TUNEL index (%) was calculated as the ratio of the number of TUNEL- positive cells divided by the total number of cells. At least eight representative fields were evaluated for each experimental group, from which an average value was calculated.

### Immunohistochemistry

Nonspecific binding was blocked with 5% normal goat serum. Then the slices were incubated overnight with anti - MMP2 antibody and anti - TIMP2 antibody. Staining was visualized with the streptavidin - perosidase reaction using diaminobenzidine (Boster Bio - engineering Limited Company, Wuhan, China) and the images were analyzed by staining densitometry using Adobe ImageReady 7.0.1 software (Adobe Systems, San Jose, CA).

### Plasma Concentration of Apelin

Apelin concentration was determined using the apelin-12 ELISA assay kit (Phoenix Pharmaceuticals INC, Belmont, CA, USA), following the manufacturer’s instructions. The antibody used in this apelin assay cross-reactivity 100% with rat apelin-13 and apelin-36.

### Cardiomyocyte Isolation and Culture

A Langendorff perfusion method according to the criteria adapted as previously described [20]. The heart was rapidly cannulated via the aorta attached to a Langendorff perfusion apparatus and perfused with Krebs Henseleit (KH) buffer containing 1 mM Ca^2+^ for 5 minutes in a retrograde manner. Then a low-Ca^2+^ solution was changed to perfuse 5 minutes followed by 1 mg/ml collagenase buffer for 10 minutes. The temperature remained 37°C unchanged throughout the perfusion. The heart ventricles were cut into small sections and incubated with collagenase buffer in a thermostat water bath tank for 3 minutes at 35°C. The cardiomyocytes were collected by centrifuging with 400 rpm at room temperature for 1 minute and then cultured as previously described [21]. After 48 hours culture, the supernatant and cardiomyocytes were collected by centrifuging for use.

The article "The Complex Regulation of Tanshinone IIA in Rats with Hypertension-Induced Left Ventricular Hypertrophy" was retracted in 2024. Reasons: duplicated images; duplicated data; overlap with earlier publications; original data or images not available.

### Assessment of Oxidative Stress

The activity of malondialdehyde (MDA) and superoxide dismutase (SOD) in cultured cardiomyocytes was measured by use of the commercial kit (Jian-Cheng Biochemical Engineering, Nanjing, China). The absorbance was detected at 532 nm and 550 nm with use of a spectrophotometer (UV-2450, Shimadzu, Kyoto, Japan) separately.

### Myocyte Supernatant Markers of Cardiac Fibrosis

TGF-β1 and bFGF were measured with ELISA kits used according to manufacturer’s instructions (R&D systems, Minneapolis, Minnesota, USA). Values were normalized to a standard curve.

### Western Blot Analysis

The proteins were extracted from cultured cardiomyocytes, using the Micro BCA Protein Assay Kit (Pierce, Rockford, IL, USA) to quantify protein concentrations as previously described [22]. Protein was then used for Western blotting with primary antibodies against Bax, Bcl-2, Caspase-3, Foxh1, c-Myc, p-Smad3 and APJ. All images were captured and analyzed by the Gene Genius system (Syngene, Cambridge, United Kingdom).

### Statistical Analysis

All the data were presented as mean ± standard deviation. SPSS 13.0 Software was used for the data analysis. Student’s t-test was applied for the statistical significance between the sham and H-LVH (5%GS) group. A repeated measure ANOVA with Bonferroni’s post test was used for comparison among four groups of H-LVH rats. P<0.05 demonstrated statistical difference.

## Results

### General Characteristics and Echocardiography Parameters

Twelve weeks after operation, remarkable increase was noted in LV Mass, LV Mass/BW, mSP, IVSd and LVPWd in the H-LVH (5%GS) group compared with those in the sham group (P<0.05). For the above parameters except mSP, significant decrease was observed after treatment of tanshinone IIA in H-LVH rats than those of the 5%GS group (P<0.05, Table 1). Blood pressure was observed at two weeks intervals following tanshinone IIA therapy. But tanshinone IIA had no significant effect on pressure compared with control group (P>0.05, Fig. 1). At last, we selected the pressure before the animals sacrificed to illuminate that the inhibition of tanshinone IIA on myocardial hypertrophy was blood pressure independent. HR, FS (%), LVIDd and EF (%) in both sham and H-LVH rats were not significantly different throughout the entire experiment.

The article "The Complex Regulation of Tanshinone IIA in Rats with Hypertension-Induced Left Ventricular Hypertrophy" was retracted in 2024. Reasons: duplicated images; duplicated data; overlap with earlier publications; original data or images not available.

**Figure 1:** Systolic blood pressure in sham-operated rats (Sham) and hypertension-induced left ventricular hypertrophy (H-LVH) rats treated with 5% glucose injection (GS) or tanshinone IIA (Tan) was observed via noninvasive tail cuff (N = 8 per group). Four weeks after clipping, blood pressure was observed at two weeks intervals for eight weeks.^ #^P<0.05 compared with sham group.

**Table 1:** General characteristics and cardiac function and remodeling.

		H-LVH			
	Sham	5%GS	Tan (5)	Tan (10)	Tan (15)
Parameter	(n = 8)	(n = 8)	(n = 8)	(n = 8)	(n = 8)
HR (bpm)	386.4±40.8	410.7±42.5	403.9±38.9	421.5±35.1	411.0±43.6
LV Mass/BW (mg/g)	2.15±0.24	2.93±0.31#	2.84±0.25	2.69±0.27	2.36±0.34*
mSP (mmHg)	105.2±2.7	215.2±4.2#	207.5±3.8	212.8±4.5	216.6±4.1
IVSd (mm)	2.1±0.06	2.8±0.04#	2.7±0.04	2.5±0.05	2.3±0.06*
FS (%)	36.9±2.0	37.7±2.8	37.1±2.4	38.9±2.5	40.0±3.4
LVIDd (mm)	7.1±0.5	6.8±0.4	7.0±0.6	7.3±0.4	7.1±0.6
LVPWd (mm)	1.7±0.04	2.7±0.06#	2.5±0.06	2.1±0.05*	2.0±0.04*
EF (%)	74.7±4.2	72.8±4.5	74.5±5.1	78.0±3.7	77.9±3.9

# P<0.05 compared with sham group.

*P<0.05 compared with 5%GS group.

### Effects of Tanshinone IIA on Cardiomyocyte Apoptosis

The percentage of TUNEL-positive cells of left ventricular tissues in the H-LVH (5%GS) group was significantly increased compared with the sham group (P<0.05). However, the percentage of TUNEL-positive cells was significantly reduced after treatment of tanshinone IIA (P<0.05, Fig. 2A and B).

**Figure 2:** Effects of Tanshinone IIA on cardiomyocyte apoptosis. (A) Representative photographs of TUNEL-stained heart sections from different groups at 12 weeks after operation (N = 8 per group). Apoptotic nuclei were identified by TUNEL staining (buffy) and normal nuclei by hematoxylin staining (blue). (B) The percentage of TUNEL-positive nuclei was calculated. For each sample, eight randomly selected areas of TUNEL-stained slices were counted. (C) Caspase-3, (D) Bax, (E) Bcl-2 protein expression and (F) Bax/Bcl-2 ratio in isolated left ventricular cardiomyocytes of sham-operated rats (Sham) and hypertension-induced left ventricular hypertrophy (H-LVH) rats treated with 5% glucose injection (GS) or tanshinone IIA (Tan) was observed by western blot (N = 8 per group).^ #^P<0.05 compared with sham group. *P<0.05 compared with 5%GS group.

H-LVH induced cultured left ventricular cardiomyocytes protein expressions of Caspase-3 and Bax and Bax/Bcl-2 ratio significantly increased compared with control (P<0.05). Bcl-2 protein expression was slightly decreased, but did not reach statistical significance (P>0.05). After treatment of tanshinone IIA for eight weeks, we found protein expressions of Caspase-3 and Bax and Bax/Bcl-2 ratio were all reduced (P<0.05). Only Bcl-2 protein expression was enhanced compared with the 5%GS group (P<0.05, Fig. 2C–F).

The article "The Complex Regulation of Tanshinone IIA in Rats with Hypertension-Induced Left Ventricular Hypertrophy" was retracted in 2024. Reasons: duplicated images; duplicated data; overlap with earlier publications; original data or images not available.

### Effects of Tanshinone IIA on Oxidative Stress

H-LVH increased MDA content and reduced SOD content in rat cultured cardiomyocytes (P<0.05). MDA levels were significantly lower in the tanshinone IIA-treated group than in the 5%GS group (P<0.05). Furthermore, tanshinone IIA treated ameliorated the inhibited SOD activity induced by H-LVH (P<0.05, Fig. 3).

**Figure 3:** Cardiomyocytes content of malondialdehyde (MDA) and superoxide dismutase (SOD) in sham-operated rats (Sham) and hypertension-induced left ventricular hypertrophy (H-LVH) rats treated with 5% glucose injection (GS) or tanshinone IIA (Tan) was observed (N = 8 per group). (A) MDA contents in rats cultured cardiomyocytes; (B) SOD activities in rats cultured cardiomyocytes.^ #^P<0.05 compared with sham group. *P<0.05 compared with 5%GS group.

### Effects of Tanshinone IIA on Cardiac Fibrosis

In the left ventricle, an increase in the interstitial myocardial collagen content was observed in the H-LVH (5%GS) group as compared with sham groups (P<0.05). However, tanshinone IIA-treated H-LVH rats exhibited a lower interstitial myocardial collagen content than the 5%GS group (P<0.05, Fig. 4).

**Figure 4:** Collagen content was observed in rat left ventricular tissues of sham-operated rats (Sham) and hypertension-induced left ventricular hypertrophy (H-LVH) rats treated with 5% glucose injection (GS) or tanshinone IIA (Tan). (A) Upper panels were stained with hematoxylin eosin. Lower panels were stained with Masson’s trichrome. They were all taken at 200×magnification; (B) Quantitative analysis of blue stained area to the total area was used to assess the cardiac fibrosis (N = 8 per group).^ #^P<0.05 compared with sham group. *P<0.05 compared with 5%GS group.

Immunohistochemical assay showed that compared with the sham group, left ventricular tissues MMP2 and TIMP2 protein expressions of the H-LVH (5%GS) group significantly rose (P<0.05). However, tanshinone IIA reduced MMP2 protein expression and increased TIMP2 protein expression in the H-LVH left ventricular tissues (P<0.05, Fig. 5A–D). MMP2/TIMP2 ratio was higher in the H-LVH (5%GS) group than that detected in the sham group (P<0.05). Interestingly, MMP2/TIMP2 ratio was reduced in tanshinone IIA-treated H-LVH rats compared to 5%GS rats (P<0.05, Fig. 5E).

**Figure 5:** Matrix metalloproteinase 2 (MMP2, A and B), tissue inhibitor of matrix metalloproteinases type 2 (TIMP2, C and D) protein expression and MMP2/TIMP2 ratio (E) in rat left ventricular tissues of sham-operated rats (Sham) and hypertension-induced left ventricular hypertrophy (H-LVH) rats treated with 5% glucose injection (GS) or tanshinone IIA (Tan) was detected by immunohistochemistry (N = 8 per group). ^#^P<0.05 compared with sham group. *P<0.05 compared with 5%GS group.

The article "The Complex Regulation of Tanshinone IIA in Rats with Hypertension-Induced Left Ventricular Hypertrophy" was retracted in 2024. Reasons: duplicated images; duplicated data; overlap with earlier publications; original data or images not available.

In response to pressure overload, increased TGF-β1 protein and decreased bFGF protein were secreted by cardiomyocytes after 48 hours culture to activate cardiac fibrosis in H-LVH (5%GS) rats (P<0.05). After tanshinone IIA treated, TGF-β1 secretion was decreased and bFGF secretion was increased significantly than 5%GS group (P<0.05, Fig. 6A and B). Our data indicated that the levels of Foxh1 and p-Smad3 were significantly increased in cultured left ventricular cardiomyocytes of H-LVH (5%GS) group (P<0.05). Compared with the sham group, c-Myc protein expression of the rats in the H-LVH (5%GS) group was significantly reduced (P<0.05). After tanshinone IIA treated, lower expression of p-Smad3 and Foxh1 and higher expression of c-Myc than that detected in the 5%GS group (P<0.05, Fig. 6C–E).

**Figure 6:** Transforming growth factor β1 (TGF-β1), basic fibroblast growth factor (bFGF), forkhead box H1 (Foxh1), p-Smad3 and c-Myc protein expression in sham-operated rats (Sham) and hypertension-induced left ventricular hypertrophy (H-LVH) rats treated with 5% glucose injection (GS) or tanshinone IIA (Tan) was observed (N = 8 per group). (A) TGF-β1 and (B) bFGF protein expression of the supernatant in rat isolated left ventricular cardiomyocytes after 48 hours culture was detected by ELISA; (C) Foxh1, (D) p-Smad3 and (E) c-Myc protein expression in rat isolated left ventricular cardiomyocytes was detected by western blot.^ #^P<0.05 compared with sham group. *P<0.05 compared with 5%GS group.

### Effects of Tanshinone IIA on Apelin-APJ System

In H-LVH (5%GS) group, our data showed that plasma apelin level decreased and APJ protein expression increased significantly than the sham group (P<0.05). Tanshinone IIA enhanced plasma apelin level and reduced APJ protein expression in H-LVH rats (P<0.05, Fig. 7).

**Figure 7:** Plasma concentration of apelin and cardiomyocytes protein expression of APJ in sham-operated rats (Sham) and hypertension-induced left ventricular hypertrophy (H-LVH) rats treated with 5% glucose injection (GS) or tanshinone IIA (Tan) was observed (N = 8 per group). (A) Plasma concentration of apelin was detected by ELISA; (B) APJ protein expression in rat isolated left ventricular cardiomyocytes was detected by western blot.^ #^P<0.05 compared with sham group. *P<0.05 compared with 5%GS group.

## Discussion

The classic paradigm of hypertensive heart disease is from asymptomatic LVH to clinical heart failure. The transition is associated with ECM remodeling [23] and elevated LV filling pressures [24], [25]. The mechanisms include not only pressure overload but also the influences of neurohormones, growth factors, and cytokines consistent with a progressive remodeling process [26], [27]. In this study, rat models of experimental hypertension were induced using the two-kidney and one clip method. This model is one the widely-used models for the study of antihypertensive effects of various drugs or medicinal plants. After the clipping of the left renal artery, this is also a model of renovascular hypertension that has a high activation of the renin-angiotensin- aldosterone system. Angiotensin II (Ang II), the effector peptide of the renin-angiotensin- aldosterone system, is a critical mediator in neurohormonal activation in hypertension [14]. It is well known that Ang II induces cardiac myocyte hypertrophy, fibroblast proliferation, collagen formation and stimulates reactive oxygen species (ROS). These variations in the multi-factorial aetiology are involved in cardiac remodeling during the development of hypertension. Previous studies, performed in vivo and in vitro, prove that tanshinone II A can prevent Ang II - induced cardiac remodeling process by several molecular biological mechanisms, such as depressing cardiac fibroblast proliferation, inhibiting angiotensin I type 1 receptor (AT1R) gene expression [28], ameliorating cardiomyocytes hypertrophy [29] and apoptosis [30]. Moreover, tanshinone II A can also down-regulate genes related to aldosterone synthesis CYP11B1 and CYP11B2 mRNA expression and inhibit aldosterone synthesis in hypertensive left ventricular hypertrophy rats [31]. Therefore, we hypothesized that tanshinone II A could ameliorate the cardiac remodeling due to its direct or indirect effects on the AngII system. The primary goal of our study was to identify the complex regulation of tanshinone IIA in rats with hypertension-induced left ventricular hypertrophy, including myocardial contractility, ECM deposition, apoptosis of cardiomyocytes and oxidative damage. The secondary goal was to investigate the paracrine factors released by cardiomyocytes to explain the cause of cardiac fibrosis from the cellular level. The cardiomyocytes of adult hypertensive rats were isolated using a Langendorff perfusion method. Because the TGF-β1 alone could not take an effect on cardiac fibrosis. Subsequently, we explored the expressions of downstream TGF-β1 pathway components.

The article "The Complex Regulation of Tanshinone IIA in Rats with Hypertension-Induced Left Ventricular Hypertrophy" was retracted in 2024. Reasons: duplicated images; duplicated data; overlap with earlier publications; original data or images not available.

Four weeks after clipping, if SBP was higher than 160 mmHg, the animals were considered hypertensive. Then tanshinone IIA was intraperitoneal administrated daily, 5% GS as the control. Blood pressure was observed at two weeks intervals following tanshinone IIA therapy. Eight weeks later, cardiac function and dimensions were assessed by using an echocardiography system. In this study, twelve weeks after operation, remarkable increase was noted in LV Mass, LV Mass/BW, mSP, IVSd and LVPWd in the H-LVH (5%GS) group compared with those in the sham group. For the above parameters except mSP, significant decrease was observed after treatment of tanshinone IIA in H-LVH rats than those of the 5%GS group. These changes of cardiac structure and function were associated with myocardial hypertrophy inhibition effect of tanshinone IIA with blood pressure independent.

Apoptosis, or programmed cell death, playd an important role in myocardial stress, including ventricular remodeling [32]. Thus, interfering with the cardiomyocytes apoptosis was considered as a key therapy target of myocardial injury [33]. Numerous signaling pathways were implicated in mediating the process of hypertrophy-induced apoptosis, such as Bcl-2 family proteins [34] and caspases. The Bcl-2 family proteins consist of pro- and anti-apoptotic members. The balance between Bax (pro-apoptotic) and Bcl-2 (anti-apoptotic) plays an important role in determination the possibility of cells to either survive or undergo apoptosis after a certain stimulus or injury [35]. Our in vivo study showed that tanshinone IIA could inhibit cardiomyocytes apoptosis as confirmed by the reduction of TUNEL positive cardiomyocytes. Activated intrinsic signal pathways might directly trigger cardiomyocytes apoptosis in H-LVH, including the up-regulation of caspase-3 activity and ratio of Bax/Bcl-2. But tanshinone IIA modified the apoptosis signal pathway in H-LVH which down-regulated the caspase-3 activity and ratio of Bax/Bcl-2. Furthermore, our study confirmed that tanshinone IIA had protective effect on cardiomyocytes through limitation oxidative stress to change the redox state.

Oxidative stress is defined as an imbalance between ROS production and removal of excess ROS [36]. The changed redox state causes contractile dysfunction and structural damage in the myocardium, leading to apoptosis at the subcellular level [37]. Oxidative stress interaction with apoptosis represents an integral part in the pathophysiology of myocardial damage. Our study revealed that tanshinone IIA decreased MDA content and increased SOD activity in cardiomyocytes of the H-LVH group. Thus, both the activation of oxidative stress and the impaired antioxidant capacity were responsible for myocardial damage together.

Apelin peptide, its C-terminal fragments could bind with high affinity to apelin receptor (APJ) and exert biological activities [38]. The orphan seven transmembrane receptor APJ, composed of 380 amino acids, is a class A G-protein-coupled receptor (GPCR) [39]. In H-LVH (5%GS) group, our data showed that plasma apelin level decreased and APJ protein expression increased significantly than the sham group. Tanshinone IIA enhanced plasma apelin level and reduced APJ protein expression in H-LVH rats. Receptor level can vary in response to different concentration of the agonist and is sorted between recycling and degradative pathways. Thus, we suggested that tanshinone IIA was capable of reducing APJ protein expression in H-LVH rats via a direct action and an indirect action on the plasma apelin level. After activated by apelin, APJ receptor had definite protective effects on relaxing blood vessels [40], enhancing myocardial contractility and inhibiting the hypertrophy [41].

The article "The Complex Regulation of Tanshinone IIA in Rats with Hypertension-Induced Left Ventricular Hypertrophy" was retracted in 2024. Reasons: duplicated images; duplicated data; overlap with earlier publications; original data or images not available.

The dynamic balance between degradation and accumulation of ECM proteins is a physiological process that takes place in heart normally [42]. ECM in H-LVH has a profound effect on the formation of fibrotic lesions by altering its abundance, composition, and spatial organization [43]. Myocardial fibrosis is a common cause of LV remodeling, which leads to diastolic dysfunction and dilated cardiac failure. MMPs are proteolytic enzymes, whereas their activity is regulated by TIMPs as their endogenous inhibitors. Thus, the balance of MMPs/TIMPs expression is emerging as critical regulator of myocardial remodeling [44], [45]. MMP2 is a gelatinase and a collagenase [46], however, the function of TIMP2 is to inhibit a number of MMPs except MMP9 [47], [48]. Fang et al. reported that tanshinone IIA treated improved cardiac function and prevented cardiac fibrosis by regulation the MMPs/TIMPs balance in a rat model of two-kidney two-clip hypertension [49]. Our study found that compared with the sham group, left ventricular tissues MMP2 and TIMP2 protein expressions of the H-LVH (5%GS) group significantly rose. However, tanshinone IIA reduced MMP2 protein expression and increased TIMP2 protein expression in the H-LVH left ventricular tissues. MMP2/TIMP2 ratio was higher in the H-LVH (5%GS) group than that detected in the sham group. Interestingly, MMP2/TIMP2 ratio was reduced in tanshinone IIA-treated H-LVH rats compared to 5%GS rats. But our echocardiographic data indicated that the cardiac function of sham and H-LVH rats was not significantly different throughout the experimental period. Thus, our data suggested that tanshinone IIA played an important role on inhibiting ECM deposition and improving cardiac remodeling.

Profibrotic cytokine TGF-β has been reported to play a central role in regulating the composition of the ECM in many tissues [18]. In the cardiovascular system, TGF-β1 has been implicated in the development of heart hypertrophy and heart failure, associated with increasing in both cardiomyocyte growth and intercellular fibrosis [50]. bFGF induces endothelial and smooth muscle cell migration and proliferation [51], and linkage to the development of heart hypertrophy [52]. To further assess the influence of ECM-dependent paracrine mechanisms, we determinated the supernatant levels of TGF-β1 and bFGF 48 hours after cardiomyocytes cultured. As performed in this study, in response to pressure overload, increased TGF-β1 protein and decreased bFGF protein were secreted by cardiomyocytes to activate cardiac fibrosis in H-LVH rats. But after tanshinone IIA treated, TGF-β1 secretion was decreased and bFGF secretion was increased significantly than 5%GS group. bFGF is capable of suppressing TGF-β1-induced fibroblast differentiation [53] and limiting progressive fibrosis [54]. TGF-β1, after binding to its receptors, activated downstream mediators that leaded to classic Smads signaling pathways. Afterwards, phosphorylated complex of Smad 2/3 formed a higher-order complex with Smad4 which was subsequently transported into the nucleus. Smad-partner combination targeted a particular subset of genes and recruited transcriptional co-repressor c-Myc, by association with Foxh1 participated as a Smads cofactor which made Smads reach target gene specificity and target specificity [55]. Other investigations have suggested that tanshinone IIA could inhibit myocardial hypertrophy in LVH rats. The underlying mechanism might be the down-regulated expression of AT1R mRNA and Smad-3, increased production of Smad-7, and blocking TGF beta1/Smads signal pathway [56]. Our data indicated that the level of p-Smad3, a downstream receptor-regulated Smad (R-Smad) of TGF-β1 signaling, was significantly increased in the hearts of H-LVH rats. Higher expression of Foxh1 and lower expression of c-Myc resulted in higher activity of the transcription of Smads dependent genes. After tanshinone IIA treated, lower expression of p-Smad3 and Foxh1 and higher expression of c-Myc inhibited Smads induced transcriptional activation. Thus, we suggested that tanshinone IIA might provide additional beneficial effects on suppressing structural remodeling through regulating the paracrine factors released by cardiomyocytes and the TGF-β/Smads signaling pathway activity.

The article "The Complex Regulation of Tanshinone IIA in Rats with Hypertension-Induced Left Ventricular Hypertrophy" was retracted in 2024. Reasons: duplicated images; duplicated data; overlap with earlier publications; original data or images not available.

In conclusion, LVH is associated with high risk of clinical events including cardiovascular death, myocardial infarction, and stroke. However, the pathway from hypertension to LVH is not unidirectional. In search of an ideal cardio-protective agent to reduce remodeling and improve LV dilatation and systolic dysfunction, tanshinone IIA emerged as powerful candidate. Our in vivo study showed that tanshinone IIA could improve heart function by enhancing myocardial contractility, inhibiting ECM deposition, and limiting apoptosis of cardiomyocyte and oxidative damage.

## Perspectives

This study investigates tanshinone IIA as a definite protective agent for improving cardiac function in hypertension rats. The molecular mechanisms responsible for cardio-protective effects of tanshinone IIA mainly contained four balance systems, MDA/SOD, Bax/Bcl-2, MMP 2/TIMP 2 and TGF-β 1/bFGF, which may be new specific biological targets for the treatment and control of progressive cardiac dysfunction.
